The article "Application of Convolution Neural Network (CNN) Model Combined with Pyramid Algorithm in Aerobics Action Recognition" was published in 2021. Journal: Comput Intell Neurosci.

# Application of Convolution Neural Network (CNN) Model Combined with Pyramid Algorithm in Aerobics Action Recognition

**DOI:** 10.1155/2021/6170070

**Published:** 2021-09-11

**Authors:** Qi Liang

**Affiliations:** Guangdong University of Finance & Economics, Guangzhou, China

## Abstract

In order to realize high-accuracy recognition of aerobics actions, a highly applicable deep learning model and faster data processing methods are required. Therefore, it is a major difficulty in the field of research on aerobics action recognition. Based on this, this paper studies the application of the convolution neural network (CNN) model combined with the pyramid algorithm in aerobics action recognition. Firstly, the basic architecture of the convolution neural network model based on the pyramid algorithm is proposed. Combined with the application strategy of the common recognition model in aerobics action recognition, the traditional aerobics action capture information is processed. Through the characteristics of different aerobics actions, different accurate recognition is realized, and then, the error of the recognition model is evaluated. Secondly, the composite recognition function of the convolution neural network model in this application is constructed, and the common data layer effect recognition method is used in the optimization recognition. Aiming at the shortcomings of the composite recognition function, the pyramid algorithm is used to improve the convolution neural network recognition model by deep learning optimization. Finally, through the effectiveness comparison experiment, the results show that the convolution neural network model based on the pyramid algorithm is more efficient than the conventional recognition method in aerobics action recognition.

## 1. Introduction

The research on Aerobics action recognition has been going on for at least ten years, and there are many contents involved. From the perspective of recognition object, it includes routine aerobics action collection [1], aerobics type algorithm recognition, and aerobics action judgment. In the conventional method of Aerobics action recognition, generally through the analysis of data sets and the in-depth study of the key characteristics of calisthenics movements, the recognition and cognition of movement judgment can be realized [2]. The core content of the aerobics action automatic recognition system is to identify the accuracy and efficiency in the process of aerobics action recognition, which is of great significance to promote the intelligent development of the combination of pyramid algorithm application optimization and convolution neural network deep learning [3].

The article "Application of Convolution Neural Network (CNN) Model Combined with Pyramid Algorithm in Aerobics Action Recognition" was published in 2021. Journal: Comput Intell Neurosci.

With the development of the human society and the improvement of production and living standards, people's living standards are no longer just satisfied with food and clothing. People begin to pursue spiritual satisfaction based on the rich materials. Especially, after the destruction of the war of the Chinese nation, under the joint efforts of the people of the country, the national efforts of the Chinese nation have achieved and the country has been liberated. The Chinese people of all ethnic groups obtained national independence after more than 100 years, and people began to pursue the improvement of material civilization. After a series of strategic decisions such as reform and opening up, economic strength has been continuously strengthened. However, the prosperity of a country is not only the rapid development of the economy but also the integrity of the whole national spirit. Only the material and spiritual development can reflect the level of a country and the overall level of the nation. Therefore, with the continuous improvement of the economic level, China has begun to formulate relevant policies to improve the spirit of the people of all ethnic groups. The country puts forward the “people-oriented” sustainable development concept, which aims to adhere to meeting the material needs and improving people's spiritual level as the core of the development concept, which can make people's material and spiritual civilization have good and fast development. Only with a better spiritual level, the overall quality of the country can have a higher improvement and make the country develop towards democracy, prosperity, harmony, and civilization, which is also a manifestation of comprehensive strength enhanced.

Based on this background, this paper studies the application method of the convolution neural network (CNN) model combined with the pyramid algorithm in aerobics action recognition, which is mainly divided into four chapters.  Section 1 introduces the research background, necessity, and chapter arrangement; Section 2 introduces the research status of the convolution neural network model combined with the pyramid algorithm and aerobics action recognition method at home and abroad. In Section 3, the neural network recognition function combined with the pyramid algorithm is constructed. According to the unique performance and difference information of aerobics action, the three-step action discrimination and judgment of aerobics action are carried out. In Section 4, the convolution neural network (CNN) model combined with the pyramid algorithm is applied to aerobics action recognition. The experimental results and errors are analyzed, and the conclusion is drawn. The proposed CNN recognition model combined with the pyramid algorithm has higher recognition rate and recognition speed.

The article "Application of Convolution Neural Network (CNN) Model Combined with Pyramid Algorithm in Aerobics Action Recognition" was published in 2021. Journal: Comput Intell Neurosci.

The innovation of this paper lies in the application of the convolution neural network (CNN) model combined with the pyramid algorithm in aerobics action recognition. This method can decompose judgment for different types of aerobics movements and can also store and classify the identified aerobics movements by combining with compound recognition function and carry out self-training deep learning, so as to achieve the rapid recognition effect of “key information recognition-CNN deep learning model accurate recognition.”

## 2. Related Works

In recent years, the research of scholars on aerobics action recognition mainly focuses on the optimization of the action recognition process, rarely through the research of the intelligent convolution neural network system and pyramid algorithm for deep optimization [4]. And, in the previous research of the aerobics action recognition system abroad, the recognition effect of the method used is poor [5]. At present, in the research results of aerobics action recognition, there are many problems such as poor recognition effect, low recognition speed, and limited application scope. Therefore, how to improve the efficiency and intelligent recognition of aerobics action recognition has become a research hotspot [6]. Scholars from the University of Texas at Austin, United States, combined with the existing pyramid algorithm to improve the process of aerobics action recognition, put forward the pyramid algorithm combined with the idea of the neural network, and used the data information in the process of aerobics action recognition to judge the dimension, so as to realize the information deep learning and high-accuracy recognition of aerobics action, but its recognition efficiency is slow [7]. Scholars from the University of Herrington in the United Kingdom analyzed the unique movements of aerobics and proposed a fast recognition method according to the distinctive movements of aerobics in the display process, but the recognition types of this method are less [8]. In order to improve the recognition speed of aerobics movements, scholars from the University of Rochester in the United States, according to the different information of different athletes in the performance process of the same type of aerobics movements, combined with image processing technology, for the same type of aerobics movements, put forward a kind of aerobics movement recognition method that can be fast and high accuracy in the aerobics athletes group [9]. Scholars from the University of Pittsburgh found that the recognition effect of current aerobics movement is related to the surrounding environment information, so a method of aerobics movement recognition is proposed to eliminate the influence of environmental noise [10]. Scholars from the University of Melbourne in Australia found that the key action recognition nodes have a great influence on the overall recognition accuracy in the process of aerobics action recognition. Therefore, combined with the pyramid algorithm, a fast recognition model of aerobics action is proposed. This recognition method has higher recognition efficiency and recognition speed than the conventional aerobics action recognition method, but it cannot make efficient use of aerobics action data and cannot conduct in-depth analysis of the data level [11]. Scholars from Kyushu University of Japan have put forward a new “face-to-face” aerobics action recognition model through the research and analysis on the performance stability and action similarity of athletes in the process of aerobics performance and verified the effectiveness of the recognition model in the process of aerobics action recognition through practical experiments on several aerobics athletes [12].

The article "Application of Convolution Neural Network (CNN) Model Combined with Pyramid Algorithm in Aerobics Action Recognition" was published in 2021. Journal: Comput Intell Neurosci.

To sum up, it can be seen that the current aerobics action recognition system and the traditional convolution neural network (CNN) model in aerobics action recognition generally have the problems of poor recognition effect, low recognition accuracy, poor stability, and low data utilization [13]. On the contrary, in the existing aerobics action recognition system, the vast majority of recognition methods can only identify a single aerobics and cannot identify aerobics with obvious differences, so they do not have intelligent characteristics [14]. And, in the process of recognition, the utilization rate and data mining effect of the obtained aerobics action data information are also very poor [15].

## 3. Aerobics Action Recognition System Based on Pyramid Algorithm and Convolution Neural Network Model

### 3.1. Application Ideas of Pyramid Algorithm in Convolutional Neural Network Model

Pyramid algorithm is also called the Laplacian pyramid fusion algorithm [16]. In the data information to be detected or processed, the effective extraction of information is realized by image registration and image fusion for different types of image information [17]. The pyramid algorithm is often used in feature extraction and classification of intelligent data information [18]. After the information is layered, the pyramid algorithm can optimize and discretize the possible optimal solutions according to different types of problems in the process of finding the optimal solution [19]. In recent years, the pyramid algorithm has been widely used in many practical problems [20]. For example, the identification process of aerobics action, the effective information extraction process of the traffic detection image, and the image analysis process of the remote sensing satellite [21]. The pyramid algorithm is mainly to help enterprises and researchers to solve the optimization of specific objectives of specific types of problems in specific scenarios [22]. Therefore, the pyramid algorithm is similar to fuzzy mathematics, topology analysis, and image processing, but it is not completely the same, and there are still obvious differences [23]. The pyramid algorithm is based on the stability judgment and reliability analysis of the type of data to be processed, according to its differentiation characteristics to complete its intelligent judgment and accurate solution [24]. In the convolution neural network model combined with the pyramid algorithm, it is based on the convolution neural network algorithm and combined with the hierarchical processing idea of the pyramid algorithm to conduct a round of pyramid structured multidimensional analysis on the data information after convolution analysis, In this way, the results obtained by the convolution neural network algorithm have higher stability and reliability [25]. Based on this, this study combines the pyramid algorithm and convolution neural network model in the construction of the aerobics action recognition method. In the process of modeling, firstly, convolution processing is carried out on aerobics action data information, and then, pyramid hierarchical analysis is combined to achieve accurate classification of different types of aerobics action data, and the internal mathematical relationship is analyzed. Finally, according to the known aerobics action dataset library, different types of data information are analyzed, and the final recognition scheme and recognition results are output.

The article "Application of Convolution Neural Network (CNN) Model Combined with Pyramid Algorithm in Aerobics Action Recognition" was published in 2021. Journal: Comput Intell Neurosci.

### 3.2. The Construction Process of Aerobics Action Recognition System

After building the application framework of the pyramid algorithm, this study will combine the pyramid algorithm to build an aerobics action recognition system. Firstly, by combining the pyramid algorithm of spire thesaurus and deep learning strategy, three characteristic parameters of Aerobics action recognition and deep learning action recognition effect are selected, and an aerobics action recognition system combining deep learning and neighborhood regression is proposed. Through the research on the analysis process, signal conversion process, and correlation analysis of the aerobics action dataset, this paper clearly analyzes the differences and correlation of different types of aerobics action in the identification process, and the construction process of the identification system for aerobics data analysis is shown in Figure 1.

In this study, the construction process of the aerobics action recognition system is divided into the following parts.

The first part is to determine the stability differences between different types of aerobics movements. The main idea is to sort according to the correlation degree between different pyramid algorithms. In the application of this model, the original professional action dataset is first stored in the matrix space with the set dimension information and then initialized. Then, according to the dimension difference of different types of data information, the characteristic value of aerobics action recognition, deep learning characteristic value, and standard degree function *Q*(*x*) are solved:

(1) $$\begin{array}{c} Q\left(x\right)={\left(P_{1}t^{5.1x}+P_{2}t^{3.2x}\right)}^{\left(P_{1}x+P_{2}x/\sigma \right)}. \end{array}$$

The low latitude data information is represented by *P*_2_, the high dimension information is represented by *P*_1_, the standard period is *t*, the learning weight is *σ*, and the standard adaptation value is *C*.

Next, in the pyramid algorithm, we need to identify and calculate the data information; then, the standard function is *Q*′(*x*):

(2) $$\begin{array}{c} Q^{\prime }\left(x\right)={\left(P_{1}t^{5.1x}+P_{2}t^{3.2x}\right)}^{\left(P_{1}t+P_{2}x/tx\sigma \right)}. \end{array}$$

The low latitude data information is represented by *P*_2_, the high dimension information is represented by *P*_1_, the standard period is *t*, the learning weight is *σ*, and the standard adaptation value is *C*. After completing the data authenticity supplement of the function, it is necessary to carry out error calibration, and the standard function after calibration is *Q*^″^(*x*):

(3) $$\begin{array}{c} Q^{\prime \prime }\left(x\right)={\left(\frac{P_{1}x^{5.1t}}{P_{2}}+\frac{P_{2}x^{3.2t}}{P_{1}}\right)}^{\left(P_{1}t+P_{2}x/\sigma \right)}. \end{array}$$

After the calibration of the standard function, it is necessary to solve the eigenvector according to the size of the eigenvector to realize the preliminary recognition and action type judgment of different aerobics actions. When the eigenvector modulus value is larger, the higher the recognition accuracy of aerobics action is, and the smaller the eigenvector is, the lower the recognition accuracy of aerobics action is. The recognition process of aerobics is shown in Figure 2.

### 3.3. The Optimization of Aerobics Action Recognition System and the Design Process of Compound Recognition Function

In order to further improve the recognition accuracy of the aerobics action recognition system, we need to optimize the above action recognition system. Therefore, the composite identification function is introduced to complete the optimization process. The composite recognition function is a binary representation of the key information (amplitude information) of the object to be identified through the multiangle coupling correlation analysis, so as to realize the reliability evaluation of its authenticity. It is the general term of a series of effective methods for the multi-index composite function. Composite function identification is a multicriteria decision analysis method combining qualitative and quantitative analysis. It is the most widely used method for decision analysis of various problems. It decomposes the relevant factors of decision problems into multiple levels and then carries out qualitative and quantitative analysis. The simulation results of the hierarchical solution process are shown in Figure 3.

The article "Application of Convolution Neural Network (CNN) Model Combined with Pyramid Algorithm in Aerobics Action Recognition" was published in 2021. Journal: Comput Intell Neurosci.

It can be seen from the simulation results in Figure 3 that, with the increase of decomposition levels, it has more reliable data stability in the process of hierarchical solution because in the convolution neural network optimization method and recognition system used in this model, with the different number of layers, the problem to be solved is identified in advance, and the comprehensive recognition target is determined. Analysis of decision-making issues involved in the form of action and aerobics changes. In this process, if there are many factors that need to be included, it is necessary to complete further identification and data extraction of aerobics actions. In this process, it is necessary to conduct diversified analysis on the authenticity of different types of aerobics actions and set up real reliable actions as standardized reference indicators.

After the completion of the above links, in the optimization process of the aerobics action recognition system, the composite recognition function is used for multidimensional aerobics action data analysis, and the diversified evaluation function is used for correlation analysis of different types of data. In the process of analyzing the correlation degree, if the dimensions of different types of data are different, the internal function expression values are different. Therefore, it shows the difference of the recognition accuracy of the aerobics action recognition system. The simulation results of the optimization process are shown in Figure 4.

It can be seen from Figure 4 that, in the three different stages, the simulation analysis of aerobics action recognition has obvious gradient difference. This is because the data dimensions and computational complexity of different levels of data types are different, so the results are obviously different. On the contrary, the simulation results are consistent with the expected differences, and the difference recognition effect of aerobics has been significantly improved. This is because in the process of deep learning recognition in Aerobics action recognition, the proposed model will adopt different calculation strategies according to the difference of different types of aerobics action. The compound recognition function *T*_*mc*_^3^(*x*) under three-dimensional strategy is

(4) $$\begin{array}{c} T_{mc}^{3}\left(x\right)=\frac{\left(m_{1}xT_{mc}^{2}+m_{2}xT_{mc}^{1}\right)}{T_{mc}^{3}}. \end{array}$$

Among them, *x* is aerobics action data and *m* is reference constant. The composite recognition function *T*_*mc*_^*n*^(*x*) under multidimensional strategy is as follows:

(5) $$\begin{array}{c} T_{mc}^{n}\left(x\right)=\frac{\left(m_{1}xT_{mc}^{n+1}+m_{2}xT_{mc}^{1}\right)}{T_{mc}^{n+2}}. \end{array}$$

Among them, *x* is aerobics action data and *x* is reference constant. The composite recognition function also needs to evaluate and test the effectiveness of recognition quantitatively and is expressed by the test function *R*(*x*), which can be expressed as

(6) $$\begin{array}{c} R\left(x\right)=1-\left|\frac{T_{mc}^{n}\left(x\right)-T_{mc}^{n-1}\left(x\right)}{T_{mc}^{n}\left(x\right)}\right|. \end{array}$$

The recognition similarity YO is found according to the recognition similarity value of the test function.  Table 1 is the standard reference value of the measurement index YO of the test function corresponding to the composite recognition function. Among them, YO3 is the recognition similarity with Bernoulli distribution under the three-dimensional index and YON is the recognition similarity with Gaussian random distribution.

The article "Application of Convolution Neural Network (CNN) Model Combined with Pyramid Algorithm in Aerobics Action Recognition" was published in 2021. Journal: Comput Intell Neurosci.

### 3.4. Convolution Neural Network Recognition Model for Aerobics Action Data Recognition Process Optimization

In the data-solving process of the aerobics recognition system based on the convolution neural network model, there is still room for improvement in the corresponding composite function recognition method. Therefore, according to the hierarchical idea of the pyramid algorithm and the coupling analysis function of the convolution neural network model, combined with the idea of the 5-dimensional pyramid hierarchical function and convolution factor, the essence of data decomposition and data fusion of the pyramid algorithm should be applied to this deep learning recognition model. In the process of identifying the aerobics action with the conventional composite function, the data are gradually stratified from the highest dimension down and verified layer by layer. The reliability of different types of data information is analyzed, and the simulation results of the analysis are shown in Figure 5.

It can be seen from Figure 5 that, after using different types of neural network algorithms to analyze the data, it shows a gradually decreasing trend with the increase of data dimension. This is because after analyzing the recognition rules, the neural network algorithm carries out multilevel data association analysis and authenticity solution. In the analysis of the optimized aerobics action recognition system, the domain of the hypothesis factor is represented by *h*(*x*), the domain of the recognition level is represented by *w*(*x*), the membership of *h*(*x*) to *w*(*x*) is represented by *v*(*x*), and the membership of the composite recognition function is expressed as follows:

(7) $$\begin{array}{c} v\left(x\right)=\frac{h{\left(x\right)}^{\alpha }+w{\left(x\right)}^{\beta }}{\alpha +\beta }, \end{array}$$

where *x* is data processing information and *α* and *β* are vertical unit dimension vectors. In the aerobics action recognition and deep learning recognition optimization system, the pyramid algorithm and convolution neural network algorithm need to be used for quantitative analysis and error discrimination of data types in aerobics action recognition, and the quantitative analysis function *H*(*x*) and the discriminant function *P*(*x*) are as follows:

(8) $$\begin{array}{c} H\left(x\right)=\frac{\beta P\left(x\right)}{\alpha h\left(x\right)+\beta w\left(x\right)},\\ P\left(x\right)=\frac{h{\left(x\right)}^{\alpha }-w{\left(x\right)}^{\beta }}{\alpha h{\left(x\right)}^{\alpha }+\beta w{\left(x\right)}^{\beta }}, \end{array}$$

where *x* is data processing information and *α* and *β* are vertical unit dimension vectors. Therefore, in order to solve the problem of large error in the process of aerobics recognition, based on the traditional aerobics action recognition, according to the convolution neural network optimization model and pyramid hierarchical solution strategy, the dimension analysis and correlation test of aerobics action data in the input system are carried out, and the function is analyzed according to different types of fitting degree. Realize the cross analysis and stability solution of aerobics action data, and the simulation results are shown in Figure 6. It can be seen from Figure 6 that, compared with the results in Figure 5, the change rule is also affected by the data dimension, but on the whole, it will not decrease with the increase of the data dimension. When the data dimension is 5, the simulation results obtained by the three methods have better recognition stability and data reliability. Therefore, the simulation results obtained by using the fitting function can improve the stability and data reliability in the identification process.

The article "Application of Convolution Neural Network (CNN) Model Combined with Pyramid Algorithm in Aerobics Action Recognition" was published in 2021. Journal: Comput Intell Neurosci.

Before optimization, the fitting analysis function *L*(*x*) and stability judgment function *M*(*x*) are equal:

(9) $$\begin{array}{c} L\left(x\right)=\sqrt{\left|\frac{x^{\alpha }+3x^{\beta }}{3\alpha x+\beta x^{\beta }}\right|},\\ M\left(x\right)=\frac{\sqrt{\left|\left(\left(x^{\alpha }+3x^{\beta }\right)/\left(4\alpha x+\beta x^{\beta }\right)\right)\right|}}{\alpha +\beta }. \end{array}$$

The optimized fitting analysis function *L*′(*x*) and stability judgment function *M*′(*x*) are

(10) $$\begin{array}{c} L^{\prime }\left(x\right)=\frac{\sqrt{\left|\left(\left(x^{\alpha }+3x^{\beta }\right)/\left(3\alpha x+\beta x^{\beta }\right)\right)\right|}}{\alpha x+\beta },\\ M^{\prime }\left(x\right)=\frac{\sqrt{\left|\left(x^{\alpha }+3x^{\beta }/4\alpha x+\beta x^{\beta }\right)\right|}}{\alpha x+\beta }, \end{array}$$

where *x* is data processing information and *α* and *β* are vertical unit dimension vectors.

In this way, while ensuring the accuracy of aerobics action recognition, it can also effectively improve the utilization rate and analysis efficiency of aerobics action data, reduce the overall analysis time, and then reduce the system discrimination error. The optimization simulation results are shown in Figure 7.

It can be seen from Figure 7 that the simulation results of the aerobics action recognition model proposed in this study have better stability and data consistency. This is because the recognition model adopts the composite function, and the common factors in this kind of function include the correlation threshold and gray fuzzy threshold factor. Therefore, in the process of aerobics action recognition, the composite recognition function has the advantages of high stability and good data consistency. According to different types of aerobics movement data information, first remove the surrounding environment information which has nothing to do with aerobics movement, zero the relevant area, and then complete the data correlation analysis. The optimized correlation analysis function *M*(*x*) and the optimized correlation function *M*′(*x*) are

(11) $$\begin{array}{c} M\left(x\right)=\frac{\sqrt{\left|\left(x^{\alpha }+3x^{\beta }/4\alpha x+\beta x^{\beta }\right)\right|}}{\alpha +\beta },\\ M^{\prime }\left(x\right)=\frac{\sqrt{\left(\left(2x^{\alpha }+3x^{\beta }/\left(4\alpha x+\beta x^{\beta }\right)\right)/\left(3x^{\alpha }-4x^{\beta }\right)\right)}}{\alpha +\beta }, \end{array}$$

where *x* is data processing information and *α* and *β* are vertical unit dimension vectors.

The article "Application of Convolution Neural Network (CNN) Model Combined with Pyramid Algorithm in Aerobics Action Recognition" was published in 2021. Journal: Comput Intell Neurosci.

## 4. Result Analysis and Discussion

### 4.1. The Design of Verification Experiment

In the process of the experiment, the movement recognition system of professional aerobics datasets in many countries is selected as the experimental object, and the sources of the relevant original experimental datasets are obtained through the network public information. Before the formal experiment of the convolution neural network recognition system combined with the aerobics action model, we need to determine the recognition strategy according to the hierarchical verification rules of the pyramid algorithm. The relevant data of the three groups of experimental results are shown in Table 2. The experimental results are shown in Figure 8.

According to the experimental results in Figure 8, the convolution neural network model combined with the pyramid algorithm has better recognition efficiency and accuracy than other intelligent algorithms in aerobics action recognition, and its experimental error rate is also lower. This is because in the process of the experiment, after the identification step, the remaining core data information will be processed by the cross vector to solve its vector inner product. According to the numerical change trend and amplitude difference, the aerobics action information in the data can be identified, and finally, the feedback processing will be carried out according to the relevance of these information. And, it is characterized and explained in the way of two-dimensional image or three-dimensional action, so it has better recognition effect on aerobics action data in the process of the experiment.

### 4.2. Analysis of Experimental Results

In order to further analyze the validity of the experimental results, after the analysis of the data types, the objectivity of the identification results needs to be further evaluated. In the experimental data of the aerobics action recognition system, the relevant experimental datasets in the pyramid algorithm are processed by MATLAB and Excel software. In this optimized recognition method, the experimental results need to be verified, and the verification results are shown in Figure 9.

It can be seen from Figure 9 that the convolution neural network aerobics recognition model based on the pyramid algorithm can promote the efficiency of aerobics action recognition, and it has better recognition stability. At the same time, it can further improve the quality of aerobics action recognition and traditional deep learning recognition optimization, and its recognition quality is also further improved. Compared with other methods in the experiment, the relative error is also reduced.

The article "Application of Convolution Neural Network (CNN) Model Combined with Pyramid Algorithm in Aerobics Action Recognition" was published in 2021. Journal: Comput Intell Neurosci.

## 5. Conclusion

Nowadays, there are some problems in the method of aerobics action recognition, such as large proportion of subjective factors and low degree of intelligence. Based on this, this paper studies the application of the convolution neural network model combined with th epyramid algorithm in aerobics action recognition. Firstly, according to the hierarchical idea and basic architecture of the pyramid algorithm, combined with the known convolutional neural network (CNN) model, an intelligent aerobics action recognition system is proposed. Secondly, this paper constructs the pyramid algorithm in the system of the compound recognition function, analyzes the conventional optimization effect recognition method in the optimization recognition, aiming at its shortcomings to improve, and uses the pyramid algorithm to deeply optimize the aerobics action recognition system. Finally, the experimental results show that the aerobics action recognition system based on the pyramid algorithm and convolution neural network model has the advantages of good speed index, high degree of intelligence, and high degree of accuracy, and the effectiveness of the system is verified by many kinds of datasets. The innovation of this paper lies in the application method of the convolutional neural network (CNN) model combined with the pyramid algorithm in aerobics action recognition. This method can make decomposing judgments for different types of aerobics actions and can also combine the compound recognition function to store and classify the recognized aerobics actions data and carry out self-training deep learning, so as to achieve the “key information recognition-CNN deep learning model-accurate recognition” fast recognition effect. But this study only considers the action recognition of aerobics dataset, without considering its application effect in specific aerobics, so we can carry out deeper research.

## Figures and Tables

**Figure 1:** The construction process of the aerobics data analysis recognition system.

**Figure 2:** Recognition process of aerobics movements.

**Figure 3:** Simulation results of the hierarchical solution process.

**Figure 4:** Different simulation results of aerobics movement recognition.

**Figure 5:** Different simulation results of aerobics movement recognition.

**Figure 6:** Different simulation results of aerobics movement recognition.

**Figure 7:** Optimized simulation results of aerobics movement recognition.

**Figure 8:** Function images of different experimental objects during the experiment.

The article "Application of Convolution Neural Network (CNN) Model Combined with Pyramid Algorithm in Aerobics Action Recognition" was published in 2021. Journal: Comput Intell Neurosci.

**Figure 9:** Verification and evaluation of experimental results. (a) Pyramid algorithm convolutional neural network recognition model. (b) Routine aerobics action recognition model.

**Table 1:** Standard reference values for optimization indicators.

*n*	1	2	3	4	5	6	7	8	9	10
YO3	0.13	0.24	0.35	0.46	0.57	0.68	0.79	0.91	0.95	0.98
YON	0.14	0.26	0.39	0.48	0.58	0.69	0.82	0.94	0.97	0.99

**Table 2:** Analysis data of 4 sets of experimental results.

Indicators and models	The first set of aerobics data	The second set of aerobics data	The third set of aerobics data
Routine aerobics action recognition model	8.2	8.4	8.1
Pyramid algorithm convolutional neural network recognition model	8.9	8.7	9.5
Convolutional neural network recognition model	8.3	8.5	8.5

## Data Availability

The data used to support the findings of this study are available from the corresponding author upon request.
